The article "A Modified ResNeXt for Android Malware Identification and Classification" was published in 2022. Journal: Comput Intell Neurosci.

# A Modified ResNeXt for Android Malware Identification and Classification

**DOI:** 10.1155/2022/8634784

**Published:** 2022-05-20

**Authors:** Marwan Ali Albahar, Mahmoud Said ElSayed, Anca Jurcut

**Affiliations:** ^1^School of Computer Science, Umm Al-Qura University, Mecca, Saudi Arabia; ^2^School of Computer Science, University College Dublin, Belfield, Dublin, Ireland

## Abstract

It is critical to successfully identify, mitigate, and fight against Android malware assaults, since Android malware has long been a significant threat to the security of Android applications. Identifying and categorizing dangerous applications into categories that are similar to one another are especially important in the development of a safe Android app ecosystem. The categorization of malware families may be used to improve the efficiency of the malware detection process as well as to systematically identify malicious trends. In this study, we proposed a modified ResNeXt model by embedding a new regularization technique to improve the classification task. In addition, we present a comprehensive evaluation of the Android malware classification and detection using our modified ResNeXt. The nonintuitive malware's features are converted into fingerprint images in order to extract the rich information from the input data. In addition, we applied fine-tuned deep learning (DL) based on the convolutional neural network (CNN) on the visualized malware samples to automatically obtain the discriminatory features that separate normal from malicious data. Using DL techniques not only avoids the domain expert costs but also eliminates the frequent need for the feature engineering methods. Furthermore, we evaluated the effectiveness of the modified ResNeXt model in the classification process by testing a total of fifteen different combinations of the Android malware image sections on the Drebin dataset. In this study, we only use grayscale malware images from a modified ResNeXt to analyze the malware samples. The experimental results show that the modified ResNeXt successfully achieved an accuracy of 98.25% using Android certificates only. Furthermore, we undertook extensive trials on the dataset in order to confirm the efficacy of our methodology, and we compared our approach with several existing methods. Finally, this article reveals the evaluation of different models and a much more precise option for malware identification.

## 1. Introduction

Malware has many different definitions specified by different scholars and researchers depending on the attack vector deployed or harm caused. However, all researchers agreed on the same meaning in general, that is, malware applications have an evil intent [1]. Malicious software (malware) is any software with malicious intent. Malicious code is designed to disrupt normal functioning, display unwanted advertising, control the user's device without their awareness or knowledge, steal or gather sensitive information, and delete or encrypt important data [2]. Unintentionally, harmful software and malware are collectively referred to as “bad ware.” The newly developed malware, which is very sophisticated, can obstruct emulators and elude deep static analysis. Malware can also be spread through metamorphic techniques such as instruction permutation, registry modification, encryption, antidebugging, multipacket, virtual machines, and code transformation. It has the capability to launch the payload intelligently to evade detection techniques [3–7]. Many new variants of malware can be generated using automation and reused development modules [8–10]. Like computer systems, malware systems have evolved enormously to be smarter, more intelligent, and more decisive. The main categories of malware are botnets, ransomware, viruses, rootkits, worms, and Trojans [10]. Malware can avoid detection by using polymorphic and metamorphic techniques [3, 11–13]. Malware developers frequently modify minor portions of the original source code in order to create new variants and avoid detection [9, 14, 15]. This makes it extremely difficult to distinguish malware variants from the same family [16, 17].

Malicious Android applications can infiltrate smartphones to be able to do anything without the user's knowledge, such as stealing information, blocking access to critical information from the device, or even mine cryptocurrency. Currently, the rate shows an incredibly high increase in Android malware samples (malicious Android apps) and their variants keep proliferating. The McAfee mobile threat report in Q1 2020 [18] announced that the size of new detected malware attacks reached 800,000 in the 4th quarter of 2019, exceeding the previous quarter of 35 million malware attacks.

Some of these attacks are not easy to detect since the attacker mimic the same normal behavior. For example, the attackers develop a new malware, named MalBus, to avoid any detection by using the original developer's Google Play account.

Moreover, the attacker can collect sensitive military and political information using scannable devices as well as target Google account login information using a phishing-style fake login page. Besides, a new Android malware family (i.e., LeifAccess), which is also known as Shopper, works by exploiting accessibility advantages to create accounts and post fake reviews on the Play Store. After installing it, it promotes click fraud without displaying an icon or a shortcut. As a result of the rising threat from an ever-increasing number of mobile malware instances and new malware families emerging, the Android ecosystem's security will be affected. In order to combat this threat and protect mobile users and systems [19, 20], many studies have been conducted to look for ways to detect and classify Android malware samples. As follows, there are many problems related to the classification and detection of malware: the problems of binary classification in which an app's malignancy is attempted to be determined, multiclass classification problems that include attempting to classify detected malicious apps into a known or unknown family, which is related to identifying malware families, and many others. So, malware researchers should be focusing their attention on the most dangerous families instead of focusing on individual malware samples or lower-risk families if samples are correctly classified and accurately characterized [19]. As a result, an effective malware family classification can assist malware analysts in identifying more malware samples by recognizing and understanding the characteristics of other malware samples in a family. On the other hand, there is a more challenging task than malware detection, which is the classification of malware families. The reason for that is that the numbers of malware samples vary extremely between different families [19–22].

Windows malware families have been the subject of several malware classification studies [9, 17, 23–25]. Due to the different structures and characteristics between Windows malware and Android malware, it is not applicable to utilize the same methodologies to categorize Windows malware families for Android malware families [25, 26]. Consequently, Android malware samples and variations have recently received a lot of attention from academics and the industry.

A recent publication [27] sheds light on the advancement of malware detection through the use of the ResNeXt model. This advancement is due to the architecture of the model, which combines the features of the ResNet and InceptionNet architectures. In addition, it requires low flops and applies the skip concept from ResNet architecture. Motivated by this fact, we proposed a modified ResNeXt model for Android malware classification. The proposed model operates on raw bytes, obviating the need for decryption, disassembly execution of code, and reverse engineering in order to identify malware. To extract the quality information, we converted the malware's nonintuitive features into fingerprint images. Seeing through malware binary, we evaluated the performance and generation of the proposed model to view the capability of discovering and extracting insights necessary for malware analysis and to pave the path for the development of effective malware classification systems.

The main contributions of this work are enumerated as follows:

- Proposes an effective modified ResNext classification network for automatically classifying Android malware families from raw malware samples. The Drebin dataset was used to test and validate the proposed system. This dataset contains 5560 applications from 179 different malware families.
- Investigates fifteen different combinations of Android malware file structures in order to classify and generate malware images. In addition, we observed that CR combination of malware image is the most suited feature for malware identification and classification.
- We extract composite features by designing a modified ResNext with a new regularization technique. In particular, we used the standard deviation of the weight matrix to create an adaptive weight decay form in order to prevent the model from taking values.

The rest of this study is organised as follows: Section 2 provides a brief background about the structure of the API files, CNN, deep residual networks, and regularization techniques.  Section 3 provides an in-depth view of the existing promising countermeasures that have been produced to monitor and detect Android malware categories. The dataset analysis, methodology, and proposed model are described in Section 4.  Section 5 discusses the experimental results and analysis, while an overall discussion of this research and the limitations are introduced in Section 6. Finally, the study' conclusion is discussed in the last section.

## 2. Background Theory

This section provides a brief background to introduce the structure of the API files and other classifiers and regularization techniques, which are applied for our classification problem.

### 2.1. Structure of APK Files

Android has become one of the most popular operating systems for smartphones. Since the Android operating system is open source, cybercriminals are attracted to using it. This section goes over the Android application, common Android malware families, Android malware analysis, and Android malware detection techniques. Generally, Android applications are mainly written using the Java programming language and then gather data and source files into an archive file called the Android application package (APK) (Android package) [28]. The APK is shared in the application market and is used for the installation of applications. However, the APK is a ZIP file consisting of multiple files, making it necessary to unzip it before use [29]. The Android APK structure is shown in Figure 1, and the details of each file and folder component are given in Table 1.

Malware families are groups of malwares with similar characteristics, behavior, and capabilities, such as stealing information from a location or a remote server, sending paid or malicious SMS messages, and so on. Malicious behavior uses the same package names as the attack for injecting a payload. In addition, the identity (signature) of a group of malwares (family) can be determined by repeating the use of package names (or other common characteristics) [19]. The most common malware families are given in Table 2 [18].

A significant amount of time is required to manually create features throughout the Android package (APK) structure for Android malware family classifications [3, 4, 30, 34, 35]. These safety mechanisms require significant computer resources, and their deployment in a restricted smartphone environment is challenging [31]. Android malware traces have been studied through classes.dex (CL), resource (RS), manifest, and Android application certificate (CR) files. Malware detection technology, as well as malicious code, have both been developed over time. It is necessary to analyze malware in order to be able to detect it. There are several methods for analyzing and classifying malware, including static, dynamic, hybrid, visualization (image), and audio [32, 33]. Static analysis and classification are the most common methods. Antimalware signatures and behavioral techniques such as static and dynamic analyses are the most important techniques for identifying malware. Intelligent malware, on the other hand, employs dynamic analysis in conjunction with antiemulation technology [28, 31, 36]. In order to use dynamic and static techniques on such files, a significant amount of manual effort or human intervention is required. To reverse engineer or analyze an application, it is necessary to have prior knowledge of the domain [29, 37–40].  Table 3 provides a comparison between two types of analysis, which are static and dynamic analyses.

However, the dynamic approaches experienced with false-positive rates can hinder their wild deployment in real applications. In general, dynamic malware detection is resilient to metamorphic and polymorphic malwares. However, they are slow, resource-consuming, and vulnerable due to the limitation of code reachability. Hence, they may be including a false positive rate. In practice, the weight value for each feature of an application indicates how significant the feature contributes to the classification result in the model pool that participates in the weighted voting that derives the classification result for the application. So, the abnormal feature values in terms of sensitive access might cause some benign apps to be falsely classified as malware. Thus, we can see the dynamic methods are not sufficient and scalable to trace many malicious apps. Moreover, since malware coders have more experience using traditional detection and classification techniques, it will be easier for them to create new malware that can circumvent the current security mechanism. For this reason, researchers have been working for the past few years to develop a new, faster method of automatically detecting, visualizing, and classifying malware. In 2011, Nataraj et al. [24] proposed a completely new approach to malware visualization and analysis using the image processing concept. This is done by visualizing the malware as binary images, extracting its features, and then classifying it. However, the system classifies malware into different families based on whether it has the same visual features, similar texture, and similar structure as malware belonging to another family [2]. This technique overcomes several limitations inherent in static and dynamic analyses. This motivates us to focus on visual-based analysis as it provided a new direction for deploying convolutional neural network (CNN) algorithms for the purpose of detecting malicious software effectively. The images generated by the visualization approach have a variety of layouts, styles, and forms. Thus, malware images have distinct visual similarities and characteristics that set them apart from benign images, which are distinguished by a variety of distinct stripes. These striking distinctions in the visual characteristics of acquired benign and malware images help us classify them according to their families.

### 2.2. Convolutional Neural Network (CNN)

CNN is one of the neural network (NN) algorithms widely used for computer vision. However, in the traditional NN, the hidden layers are fully connected with each other, which significantly increases the number of training parameters, and this can increase the complexity of the classifier. The CNN produces the concept of parameter sharing in each layer to solve the limitations of the traditional NN and reduce the explosion of weight vectors. The weight sharing concept of the CNN can reduce the computational cost and the training time of the model classifier compared to the other DL models. The CNN is constructed from three core layers, i.e., convolution, pooling, and fully connected layers [48]. The simple architecture of the CNN is shown in Figure 1. The convolution layer is produced as a result of the linear operation of the kernel or filter with the previous output layer. The Relue activation function is widely used in the CNN to increase the degree of nonlinearity and to remove also all negative values of feature maps. The CNN can include more than a convolutional layer. The first layer is used to capture the simple features such as corners or edges. While, the higher layers are mainly used to learn the high-level features. The CNN does not only have the capability to extract the discriminatory features from the input data but can also reduce the spatial size of the convolved feature through the pooling layers. The CNN is implemented in several available architectures, such as ZFNet [49], ResNet [50], GoogLeNet [51], VGGNet [52], AlexNet [53], and LeNet [54]. Motivated by the success of the CNN in various application domains, we utilize the CNN for Android malware detection. The parameters' sharing and the concept of dimensionality reduction are the factors that inspired us to use the CNN for the detection problem.

### 2.3. Deep Residual Networks

In 2016, Microsoft Research Lab [55] released the deep residual network to solve the inherent problems of traditional deeper networks. The traditional models are more difficult to train and exposed to the degradation problem (of training accuracy). Adding new layers to the deeper networks not necessarily improves the training accuracy. In most cases, the accuracy becomes saturated and will degrade rapidly with increasing of the network depth, and this can lead to high training errors. On the other hand, the deep residual network works to overcome the aforementioned limitations by using the residual blocks. The simple structure of residual building block is shown in Figure 2.

The potential of this type of networks lies on the concept of “skip connections” to improve the accuracy of the models. Instead of the consecutive connections of the layers in the neural network, some of the layers are skipped and feed the output of one layer as the input to the next layers. The residual blocks are stacked together in a sequential way to consist the residual. The identity mapping of deep residual is descried according to the following formula:

(1) $$\begin{array}{c} X_{i+1}=X_{i}+F\left(X_{i},W_{i}\right), \end{array}$$

where *F* is the residual function, *W*_*i*_ is the wight parameters of the block, and *X*_*i*_ and *X*_*i*+1_ represent the input and output of the *i*^th^ unit in the network. In recent days, the deep residual approved its robustness in several computer vision applications. Motivated by its successfully achieved results in different tasks, we also utilized deep residual in this article for Android Malware detection.

### 2.4. Regularizer Technique

#### 2.4.1. Regularization: A Method of Controlling the Model from Complexity

One of the big challenges in machine learning is how to build a more robust model that can perform effectively in the training data and the new testing data as well. However, the overfitting is one of the significant problems that can hinder the normal operation of machine learning techniques. The model can perform very well during the training, but unfortunately, it performs very poor in the new testing samples, which eliminates its wild implementation for zero-day attacks. The reason behind that returns to the complexity of the training model, resulting from large number of training parameters. As a result, the model can learn the noise in the input data as specific features to discriminate between different attack classes. To eliminate this problem and reduce the error of the prediction model, we can use regularization techniques. The key idea behind the regularization methods is to penalize the model by dropping some of its weight parameters, and this can increase the model's performance on unseen data detection. There are many several techniques widely used for the regularization process. L1 and L2 are the most two popular regularizer methods and comprehensively used in the domain area of machine learning [56]. In the following subsections, we will discuss these two methods in detail.

#### 2.4.2. L1 or Lasso Regularizer

In the L1 regularizer, the absolute value of the magnitude is added to the new loss function. Penalizing the model with the absolute value will make the weight parameters of the insignificant features to reach to zero. As a result, these features will be ignored totally from the model training, i.e., are not contributing any more for the classifier's boundaries. So, we can find the L1 regularizer is widely used for feature selection purposes to selectively reduce or eliminate unnecessarily features [56]. The L1 regularizer is denoted mathematically as follows.

(2) $$\begin{array}{c} \lambda \sum_{i=1}^{n}\left|w_{i}\right|, \end{array}$$

where *λ* is the new hyperparameter used for regularization, *n* represents the number of features in dataset, and *w* gives the weight values of each feature.

#### 2.4.3. L2 or Ridge Regularizer

In the L2 regularizer [56], we added the square value of the magnitude to the new loss function instead of the absolute value like in L1. Thus, the weight of less important features will reach close to zero but never reach digit zero itself, i.e., the weight matrix will remain greater than zero. L2 regularizer provides better performance with low loss compared to L1. Since, it considers all features during the training process [57]. The mathematical notation of the L2 regularizer is discussed in the following equation:

(3) $$\begin{array}{c} \lambda \sum_{i=1}^{n}w_{i}^{2}. \end{array}$$

The *λ* is the hyperparameter parameter and used to impose an additional penalty on the corresponding weight values and *n* and *w* represent the number of features and the coefficient value of each feature, respectively.

#### 2.4.4. New Regularizer

As we explained in the aforementioned section above, the L1 regularizer is widely used for feature selection, while the L2 regularizer gives less importance to less significant features. However, both regularizers have substantial drawbacks and inherit some limitations, which hinder their broad use to detect zero-day threats. Unfortunately, L1 and L2 regularizers do not take into account the relationship between entries in a weight matrix. In other words, they only deal with individual weight values. However, any change in the feature attributes, even a small change, can cause a big difference in the model performance. To solve this problem, we developed a new regularizer method (SD-Reg) based on the standard deviation to efficiently deal with the weight values' dispersion, i.e., the SD-Reg regularizer restrains the learning model of using a diapered range of weight space. It works to create a weight-decay adaptive form by considering the standard deviation of a weight matrix and multiplies it by *λ* parameter to obtain its regularization term.

It is shown in equations (3)–(5) how to formulate the new regularizer.

(4) $$\begin{array}{c} \lambda \sigma \left(w\right), \end{array}$$

where *σ* indicates the standard deviation of the following weight values:

(5) $$\begin{array}{c} \sigma \left(w\right)=\sqrt{\frac{1}{nk}\left\{\sum_{i=1}^{nk}w_{i}^{2}-\frac{1}{nk}{\left(\sum_{i=1}^{nk}w_{i}\right)}^{2}\right\}}. \end{array}$$

For each row of the weight matrix, there are *k* rows; each row corresponds to an individual weight. Whereas, *σ* stands for the standard deviation's weighted averages. *n* is the number of columns in each *i*^th^ row of the weight matrix, which is controlled by the parameter *λ*. The weight vector has a length of *n*. In our case, the loss function is

(6) $$\begin{array}{c} \min_{w}\left\{f\left(X,y:w\right)+\lambda \sigma \left(w\right)\right\}. \end{array}$$

Thus, the standard deviation of *w* is used to minimize the loss function for *w* in order to select a specific range of values.

## 3. Literature Review

Recent years have witnessed a significant increase in the number of Android malware cyberattacks. On the other hand, there are substantial efforts by malware researchers and cybersecurity scholars to develop new reliable techniques in order to identify and mitigate the frequent development of these attacks. As a result, the automated Android malware detection (AMD) to deal with this critical cybersecurity challenge has increased too and cannot be neglected.

On the other hand, comprehensive AMD approaches have witnessed a significant increase in the use of ML and DL techniques to ensure the security of the Android ecosystem. This section represents the most widely employed ML and DL approaches for Android malware detection.

### 3.1. Malware Detection Based on ML

Several ML algorithms such as logistic regression (LR), random forest (RF), k-nearest neighbor (KNN), and support vector machine (SVM) have been used for Malware attack detection.

In [58], three ML classifiers, namely, KNN, RF, and DT were used for AMD on APK samples, which consisted of 300 benign samples and 183 malwares. The Dalvik opcode was extracted from the classes.dex file and then converted into an 8-bit grayscale image. The GIST descriptor was used later to extract the input attributes from the created images. The experimental results showed that RF provided better accuracy of 84.14%.

Li et al. [59] produced a lightweight model for AMD using the SVM algorithm on a dataset downloaded from Google Play store. The authors used less number of permissions for malware classification instead of using all the requested permissions, i.e., selected the top permissions that are more specific for benign and the top permissions for malware to build the malware detection system.

Wang and Li [60] utilized three different ML algorithms, including NB, DT and K-nearest neighbors, for AMD. The feature selection and reduction techniques were used at the first stage to reduce the number of training features and to create a lightweight model with less number of features.

In the study by Massarelli et al. [20], the dynamic analysis was used to find the resource consumption metrics, including CPU, memory, and network usage, as input features of the training classifier. The SVM was utilized to identify several Android malware families on the Drebin dataset.

Chen et al. [61] proposed TinyDroid for AMD. The authors extracted the opcode sequence from Dalvik Executable files and then used the n-gram to extract the trained features from the opcode data. Four ML algorithms, RF, KNN, SVM, and NB, were used for the classification process to identify the malicious malware from normal APKs.

However, most of the aforementioned methods mainly used feature engineering in order to find the best features of the input data. However, selecting the best features is not an easy task, since the features that can work efficiently for one malware class are not necessarily important for other classes. Besides, the input data almost has a high degree of nonlinearity, and shallow learners have a poor ability to learn the complex and nonlinear structure of the data.

### 3.2. Malware Detection Based on DL

In recent days, deep learning (DL) techniques have been conducted in several application domains, such as image processing and speech recognition [62]. The high potential of DL in several applications returns to its capability to extract the representation features from the input data automatically without any human intervention. It has the good capability to work in data, which has a high degree of nonlinearity, in contrast to shallow learners, almost experienced with high false alarms as they require hand-crafted features as input. The high performance of DL in intensive domain areas encourages many organizations and enterprises such as Facebook, Google, and Microsoft to deploy DL in various applications [63]. Researchers are also starting to leverage DL for cybersecurity tasks and malware detection as well.

Huang and Kao [64] proposed a new model, namely, R2-D2 for detecting the Android malware. The authors first obtained fixed size colored images from the classes.dex bytecode of the Android archive file. Then, different network models based on the CNN algorithm were used for the training and classification processes. A realistic dataset with more than 2 million of benign and malicious malware samples was collected in the period from January 2017 to August 2017 for the research work.

Hardy et al. [65] used the stacked autoencoders- (SAEs-) based DL model for malware detection. The model composed of two phases. In the first phase, unsupervised learning was used to extract the discriminatory features of the input data. The API calls extracted from the Portable Executable (PE) files were used as input features for the DL model. In the second stage, fine-tuning based on supervised learning was used to adapt the weights and offset vectors. A dataset collected from the Comodo Cloud Security Center is used for a comprehensive experimental study to compare various malware detection models.

Kim et al. [66] proposed an Android malware detection model using a multimodal deep learning method. Seven diverse features have been extracted from the unzipped APK, i.e., shared library, dex, and manifest files. The collected features are merged together to create a fixed feature vector. In the classification process, the DNN was used on malware samples produced from three different sources, i.e., VirusShare, MalGenome project, and Google Play app store.

Another detection approach, i.e., MalDozer was proposed by Karbab [67] for Android malware classification. The CNN with one convolutional layer followed by another softmax layer and one fully connected layer was used to detect samples of unknown malware families. The classifier approach has been applied on three different datasets, including MalGenome, Drebin, and merged datasets. While, API calls that appear in the DEX file were extracted for input attributes.

Nix and Zhang [68] investigated the CNN for Android application/malware classification. The code included within the classes.dex was examined to obtain API calls as an input attributes. The CNN approach was compared with LSTM and other n-gram-based methods on a dataset collected from the Contagio Mobile repository. The results showed that the CNN outperformed the other classifier techniques.

Suarez-Tangil et al. [3] proposed DroidSieve to classify the malware samples using a static solution. Several features have been used to identify the normal samples from the malicious malware, such as API calls, native code, invoked components, code structure, and permissions. The authors used Drebin and MalGenome datasets for their experimental evaluation. However, the reported results relied on the Drebin dataset during its large size and covered all MalGenome samples. The obtained results approved that the DroidSieve approach successfully achieved high accuracy when using resource-centered features and reducing code analysis.

Along with dynamic features derived from an application's behavioral profile, such as method calls and intercomponent communication (ICC) intents, DroidCat [69] identified and classified Android malware. Using apps that have evolved over the last nine years, it classified them with 97% accuracy. It was able to defeat attacks that targeted system calls or sensitive APIs, as well as malware samples that used obfuscation schemes. It outperformed two state-of-the-art techniques in terms of detection accuracy, using MalGenome, Drebin, AndroZoo, and VirusShare datasets [70]. It relied on a variety of machine learning algorithms, including SVM, Naive Bayes, and RF. The RF with 128 trees outperformed all other methods. Because the dynamic malware analysis technique proposed by Ficco [71] is composed of a combination of generic and specialized detectors that are used throughout the analysis process, it is resistant to specific evasion techniques. To address malware evolution, the proposed technique utilized an alpha-count mechanism to investigate the effect of varying the length of the observation time window during run-time on the accuracy and speed of detectors. He demonstrated the technique's efficacy using data from 27 DREBIN families. Additionally, a second validation dataset, spanning the period June 2013 to March 2014, was used as a validation dataset taken from the VirusShare dataset.

In this research work, we propose an accurate and automated vision-based AMD model to deal with the critical cybersecurity challenges, which are difficult to ignore. A fine-tuned DL-based CNN algorithm is developed to efficiently detect malware attacks on Android OS.

On the Drebin dataset, we test several combinations and compare our approach to some state-of-the-art works, such as LeNet, Inception V3, ResNet50, Vgg16, EfficientNetB0, and SARVOTAM. All these methods are considered 2D convolution filter-based models. Also, we conduct extensive experiments and include the basic-1D-CNN with single and multistreams in our computations. The results indicate that the proposed ResNeXt achieved significant results in terms of accuracy and F1-score. In addition, the extensive computations of the ResNext model are significantly lower since it requires a smaller number of features to be analyzed compared to other methods. As a result, the modified ResNext demonstrates its effectiveness by quickly distinguishing Android malware from benign apps with the fewest recorded errors.

## 4. Materials and Methods

This section describes the methodology and the used dataset for our proposed model. The architecture and detailed explanation of the learning model are discussed in detail, considering the file size and other used parameters for the model tuning.

### 4.1. Dataset

Most of the studies that have been published between the periods of 2014 and 2020 use the Drebin dataset for training and evaluating their developed models. It is considered one of the most widely used datasets for malware family classification purposes [21]. So, for that reason, it is used in this experiment setup. The Drebin dataset has the most popular Android malware families, which were collected in the period between August 2010 and October 2012. It contains more than 5,560 files belonging to 179 special malware families like Fake Installer, GoldDream [72], GingerMaster [73], DroidKungFu [74], and many others.  Table 4 provides the outlines of different malware datasets that have been used by the research community.

### 4.2. Transforming Malware APK into Images

The fundamental files considered for visualization in APK are classes.dex, resources, manifest, and certificates. In this work, these four types from the malware APK files are employed to extract the malware images, which are used for our model training.

First, the binaries are transformed into 8-bit vectors, and in the next stage, these vectors are converted to grayscale images. The detailed procedure is discussed. Initially, a malware substring consists of a sequence of numerous substrings where each substring is 8-bit long and is called a pixel. The 8-bit substring is converted to a decimal number in the next step, ranging from 0 to 255. Furthermore, all the malware substrings were transformed into a one-dimensional vector and converted to a two-dimensional matrix of a specific width. We called it a “malicious code matrix.” This matrix is considered the two-dimensional grayscale image. The conversion process of APKs to grayscale images is shown in Figure 3. The width of the images was fixed based on the size of the APK files given in Table 5. Hence, the height also depends on the file size. CNN-based models require inputs to be of the same shape. Therefore, instead of trying varying sizes of APK files, we use the dimensions proposed by [26]. The main reason behind the chosen sizes is to retain as much information as required along with keeping the size compact. However, it is empirically decided by [17, 26]. Therefore, to avoid the trial-and-error method for finding the proper sizes, this work follows their proposed procedure. A complete APK can be represented by grayscale images with an underlying structure that follows certain divisions. Fifteen different file structure combinations were used to generate the Drebin Android malware images, each containing at least one image of a distinct malware family. Some images constructed from the files are shown in Figure 4. Classes.dex (CL), AndroidManifest (AM), certificate (CR), and resources (RS) are among the files included.

### 4.3. Proposed Model

In this work, we use the same ResNeXt classification model, which was proposed by Xie at el. [27] in order to categorize malware families. The basic idea behind ResNeXt is to use an aggregated residual block instead of the basic residual block. This strategy is called ”split-transform-merge,” and it was implemented in the inception architecture [27].

The inner product of a synthetic neural network is the weighted sum of the primary neurons in each layer, which is calculated for each layer separately. When viewed through the lens of equation (7), the inner product can be thought of as a type of aggregate transformation.

(7) $$\begin{array}{c} \sum_{i=1}^{D}w_{i}x_{i}, \end{array}$$

where *w*_*i*_ represents the filter weight for the *i*^th^ channel of the neuron, and *x*_*i*_ describes the D-channel input vector of the neuron.

A more inclusive function, which can perform as a network itself, has been developed by Xie at el. instead of a simple aggregating transformation [27]. They demonstrated aggregated transformations as

(8) $$\begin{array}{c} F\left(x\right)=\sum_{i=1}^{C}t_{i}\left(x\right), \end{array}$$

where *t*_*i*_(*x*) is an arbitrary function. Analogous to a simple neuron, here *t*_*i*_ projects *x* into an (optionally, low-dimensional) embedding and then transforms it. *C* represents the size of the set of transformations to be aggregated, while Xie at el.' study used *C* to represent the cardinality. Their study claimed that the dimension of cardinality can control great numbers of complex transformations.  Figure 5 [75] shows 32 cardinality blocks of ResNeXt.

(9) $$\begin{array}{c} y=x+\sum_{i=1}^{C}t_{i}\left(x\right). \end{array}$$

The aggregated transformation in (8) serves as the residual function, as shown in (9).

ResNeXt is designed using ResNet's skip concept and cardinality with better accuracy than a wide and deep network. In experiments using the ImageNet dataset, ResNeXt outperformed existing models in terms of accuracy. Due to these advantages, we utilize the ResNeXt model for malware image classification. The architecture of ResNeXt-50 is shown in Figure 6.

A new regularization technique was incorporated into our model in order to control individual weight values and the relationship between weight matrix entries. This is done by taking the weight matrix's standard deviation and multiplying it by *λ* to create an adaptive weight decay form. Thus, the regularizer prevents the learning model from taking values from the weight space that are too widely distributed. In fact, the new regularizer has been extensively tested on various tasks with different datasets and proved to be more effective than other regularization methods [57, 76–80].

Our model uses the new regularizer technique to control the relationship between entries using weight values from the weight matrix. To create a weight decay adaptive form, we multiplied the standard deviation of the weight matrix by *λ*. This reduces model complexity by removing unnecessary data and keeping only data that are useful for classification. The explained regularizer was tested extensively in different domains, including computer security, and provided better performance than the other regularization techniques.

## 5. Results

In this section, we briefly discuss the experimental setup and explain the classification results of the proposed approach.

### 5.1. Classification Module Training and Validation

In this research, we used the Drebin dataset with a focus on the top 20 malware families as follows: BaseBridge, Plankton, DroidDream, SMSreg, FakeInstaller, OpFake, SendPay, FakeRun, Imlog, FakeDoc, ExploitLinuxLotoor, Iconosys, DroidKungFu, Adrd, Glodream, Gappusin, Kmin, MobileTx, GinMaster, and Geinimi.  Table 6 provides Drebin malware class combinations and associated instances. The modified ResNeXt has 50 layers except for the input layer and the fully connected layer. 48 of the 50 layers are divided into 16 blocks. Each block contains three layers, with a total of 32 cardinalities.

### 5.2. Experimental Setup

In this work, all experiments have been executed using Python programming language. Several machine learning and deep learning libraries such as Keras and TensorFlow are used to build the ResNeXt model.

The simulations were run on a system with 20 GB of RAM and an Intel® CoreTM i3 processor, as well as an NVIDIA GeForce GTX 1080ti graphics processing unit with a frame buffer of 11 GB.

### 5.3. Experimental Results and Analysis

In our work, the modified ResNext model with an embedded new regularization performed well for approximately 100 epochs. The simulation results were recorded for the Drebin dataset after converting the attributes of raw malware binary executable files to grayscale images. We compared our observed performance measures with various state-of-the-art models, which indicates that the performance of our model is higher (Figure 7). The evaluation is compared for various combinations of the image types as given in Table 7.

The highest accuracy is achieved for the CR combination, as given in Table 7. As a result of the observations and simulation results, it is clear that the maximum amount of relevant information about malicious types is contained in the CR file, resulting in satisfactory classification performance. Apart from classification measures, Table 8 provides a time-based comparison for each combination used in the study and the number of images processed per second that belong to the corresponding class. The relative execution time is within a satisfactory range, which makes it possible to use it in real-time applications.

Thus, after training the model with high-quality classification measures, it can be used for testing in various applications. As given in Table 8, the average processing time for a single image is comparable to previous work [26]. Consequently, once integrated and deployed in software systems, the model's execution performance will be the same as the state-of-the-art method.

The new regularized technique was implemented in order to control individual weight values as well as the relationship between weight matrix entries in order to eliminate unnecessary data while selectively using only data useful for classification. This demonstrates the effectiveness of our model in extracting better features while also maintaining a reasonable overall running time. The detailed confusion matrix for the top 20 malware families is given in Table 9.  Table 10 provides the results of family-specific classifications for the original ResNeXt and our modified ResNeXt. As observed, the new regularization method was adaptive in order to avoid overfitting and to improve the CNN's ability to predict whether a new observation of the data was not trained on the model. As a result, it enables a more adaptable method of weight loss. As a result, the regularizer prevents the learning model from using global values from the weight space as input. This reduces the complexity of the model and removes unnecessary data, while keeping only the data that are useful for classification. As shown in Figure 8, the proposed model outperformed all the other methods of family-specific classification in terms of F1-score.

### 5.4. Malware Family Classification Performance Evaluation

It has recently become a problem for machine learning-based malware classifiers to deal with the evolution of malware, which changes its malicious behavior over time, resulting in the deterioration of the classifiers. It has been suggested that deterioration [20, 22] and model aging [17, 21] are better terms to describe this issue of long-term sustainability. Sustainability is defined as the ability of the classifier to sustain its capabilities over time without frequent retraining. Recently, the sustainability challenge associated with machine learning-based malware detection has been discussed, but with limited investigation depth and solutions.

In the same context, the authors in [20, 22] proposed and compared sustainability metrics with the five most recent Android malware detectors. Another study [81] outperformed five detectors in sustainability by employing a new behavioral profile for apps. In particular, the authors proposed DroidSpan, which surpassed the five detectors in terms of sustainability. However, their study was limited to malware detection and did not include any discussion of malware family classification. DroidEvolver [82] used a model pool with five linear online learning algorithms and delayed classifiers to perform the necessary updates. APIGraph [21] used API semantic similarity from an Android API relation graph to improve the latest malware classifiers. Therefore, we propose a modified ResNext-based classification network with new regularization for Android malware family classification. Each Android application is distributed via an Android application package (APK). An APK contains multiple folders and files, each of which contains multiple sections; an APK contains multiple folders and files; and an APK contains multiple sections. Among other files and sections, we pay close attention to the AndroidManifest.xml file (AM), classes.dex file (CL), and the certificate files included with each malware sample (CR). As a result of these sample characteristics, we chose the ResNeXt block because of its simplicity and performance. Following that, we modify ResNeXt to include a distinct block for each component (section or file) of a malware sample in order to account for the differences in characteristics between the components. A new regularization technique is utilized to improve the efficiency of malware family classification by extracting discriminatory features from the malware sample. This enables us to ultimately classify malware samples according to their correct families.

The modified ResNeXt model is divided into two distinct phases: training and testing. During the training phase, it builds a prediction model using a set of labeled samples from the Drebin dataset. Then, the trained model is used to classify samples from the Drebin and AMD datasets during the testing phase. Specifically, the primary motivation and goal for the modified ResNeXt is to demonstrate that this model can improve classification performance once trained on an older dataset and predict new patterns of malware samples from a new dataset without having to retrain on new samples.

We addressed the issue of sustainability by assessing the model's performance when it is trained on the Drebin dataset (collected between 2010 and 2012) and predicting labels for other datasets such as the AMD dataset [10] (collected between 2010 and 2016). We selected the AMD dataset because it was amassed over a longer time period than the Drebin dataset. Our experiment revealed that the feature extraction model trained on the AMD dataset outperformed the model trained on the Drebin dataset in terms of overall performance. This is because the AMD dataset contains more variation information about malware samples than the Drebin dataset, which makes it more suitable to study the evolutionary patterns of malware.

In particular, we divided the samples into three different groups, each with their own set of samples. The first group is the Drebin dataset, where we separated the malware samples from the same year into training, validation, and test sets. The goal is to assess the performance of our model with training and testing malware samples collected in the same period of time. The second group is the AMD dataset. We selected 3,460 malware samples randomly (S-AMD). By doing so, we intend to test the capability of our model in classifying apps that have never been used in training. For the third group (T-AMD), we used the entire AMD dataset, in which we utilized malware samples from different time periods than the training set. The goal is to focus on evaluating the stability of our model performance when it is trained on older datasets and predicting the labels of newer ones, spanning one to four years.  Figure 9 shows the experimental results.

In the first experiment, we compared the feature extraction model learned from the Drebin and AMD datasets (same period) to observe the performance of our model. It is clear from Table 11 that the model's generalization is better for Drebin than (S-AMD) and (T-AMD), which showed the suitability of the (S-AMD) and (T-AMD) sets in terms of containing more discriminatory features of malware samples. Next, we compared the accuracy of training and testing on the Drebin and the AMD datasets (same period and over-time). We observed that the accuracy of the Drebin dataset is better than that of the AMD dataset. This is because the Drebin dataset contains fewer malware families than the AMD dataset. In other words, the AMD dataset has sufficient variation information about malware samples, which improves the generalization performance. Thus, the generalization performance improved when the variation information of malware samples in the AMD dataset was learned.

Based on the results from Table 11, it was revealed that, even with a span of four years (the difference between Drebin and AMD datasets collection span), our model detection accuracy dropped noticeably over time from about 98% to below 80% in terms of accuracy for testing samples from year one. Over time, our model tended to be much more stable (with minimal fluctuation) in terms of detecting malware samples. It achieved an average accuracy of 87%, despite the evolution of Android malware. Despite the fact that our results are promising, we cannot claim that our model will continue to perform as well as it has in the case of future malware. The unpredictable evolution of our app in the future would also serve as a trigger for retraining our model in the future.

However, previous studies used a variety of different benchmarks casts doubt on the measurement degree of our findings' validity. As a result, despite the fact that we collected samples from a variety of sources, our datasets may not be representative of the app population during the pertinent years. Our findings and conclusions are best understood in light of the benchmarks we analyzed.

## 6. Discussion and Limitation

There are numerous benefits to utilizing DL networks for malware family classification. The DL techniques have the capability to classify data automatically without the essential requirements of some expensive processes, such as decryption or reverse engineering. However, to successfully build a lightweight classification model and to avoid the high computational cost, the size of training features must be reduced to speed up the training and detection process.

The distribution of the discriminant information is controlled via the new regularizer by constraining the weight values' dispersion. In other words, the standard deviation of the weight matrix was used to obtain the regularization term and then multiplied by *λ*. The motivation is to develop a weight-decay adaptive form that helps the regularizer prevent the learning model from extracting values from the weight space that are widely distributed. Thus, it helps the model extract features that are effective for malware family classification. Thus, the modified ResNeXt has the best classification performance among all the methods because we used a new regularization discriminant information distribution to eliminate unnecessary data and selectively use only data useful for classification.

The solutions that were representing the malicious app behaviors using dynamic features (e.g., DroidSieve) suffered from the cost of tracing runtime and scalability, while our approach incurred runtime costs for testing per second.

Additionally, the overall accomplished results for the visual grayscale images may differ from those for the visual color images. This is because color images contain more texture details and visualization features than those included in grayscale images. Also, the tested model used imbalanced Android malware samples for training and validating, so the models need to be tested on balanced Android malware samples. Thus, our proposed model avoided the computational needs of data augmentation and feature-engineering techniques. As a result, we successfully achieved better results and satisfied significant classification performance compared to other existing methods.

## 7. Conclusions

In this work, we proposed a modified ResNeXt model for the classification of android malware. The ResNeXt is utilized due to its flexibility and requirement for low flops, coupled with a new regularization technique to improve the capability of the model in the classification of android malware. In the first step, various binary malware files from the Drebin dataset were transformed into 8-bit vectors based on the substrings. In the next step, these vectors are converted to grayscale images. For classification, we adopt a modified ResNeXt with skip concept and cardinality to enhance the detection performance. Furthermore, we embedded a new regularization technique to improve the classification detection rate. Different combinations of the images were used to fine-tune the model to look for those files having the most effect on the model. From simulation results, it is concluded that the certificate (CR) is the most suited feature, containing enough information to be used for the identification and classification of malware. We reported various highest measures, including accuracy, recall, precision, and F1 measures, obtained from using the CR images. 97.07% accuracy is observed, which is the highest accuracy so far achieved by using the Drebin dataset.

For intrinsic evaluation of our DL approach, the proposed model is compared with other state-of-the-art techniques, which widely use DL for classification purposes within the Android malware family. In the future, various models can be trained and studied to adopt a less complex model, while enhancing the performance further for the malware classification problem. In addition, when malware authors distribute each malware instance in both its simple and obfuscated forms concurrently, the images between the simple and obfuscated versions are likely to differ. So, utilizing only malware images may be ineffective in this case. A possible solution to this issue is to include another feature that is resistant to obfuscation, packing, and encryption attacks and then combine it with the malware image approach, for example, the extraction of code features from native app binaries and security-sensitive APIs, including reflection-based features.

## Figures and Tables

**Figure 1:** A typical architecture of the CNN.

**Figure 2:** Residual learning: a building block.

**Figure 3:** Conversion process of APK into grayscale image.

**Figure 4:** The fingerprint images of different malware families using file sections of the Android certificate (CR), AndroidManifest (M), classes.dex (CL), and resource (RS) of an APK.

**Figure 5:** Cardinality of ResNeXt block.

**Figure 6:** The architecture of the proposed modified ResNext.

**Figure 7:** Comparison of combination classification accuracy for each model.

**Figure 8:** Comparison of family classification F1-score for each model in the Drebin dataset.

**Figure 9:** Stability comparison of classification performance on three sets.

**Table 1:** Structure of APK files.

Reference	APK folders/files	Responsibilities
[30–33]	AndroidManifest.xml	It is one of the most important files in the Android application, which stores the basic information for the applications and includes the app components, such as activities, services, broadcast receivers, content providers, and others, in addition to package information, such as permissions, package name, and app ID. It also reveals the SDK version.
	Assets/folder	The assets include the assets of an application directory, like images and files, which can be put in this folder and accessed by the asset manager object to retrieve the application assess detailed in the assets folder.
	Lib/folder	This folder contains the native code libraries. The software layer of a processor relates to a specific type of gather inside in this folder.
	META-INF/folder	This includes three main files, which are the signatures certifications, and manifest files for the APK such as MANIFEST.MF, SF, and ∗. RSA.
	Res/folder	This folder includes a description of the resources such as icons, music, images, string, resources, and layouts. These resources are not compiled in resources, arsc folder.
	Classes.dex	Dex code represents bytecode for Android applications which is generated after the compilation of the Java code. which contains multiple constructs for all classes composed like file header, string table, local variable list, class definition table, and method list and can be understandable by the Dalvik virtual machine. Any change in the dex file will affect the APK.
	Resources.arsc	This includes an application's resources in a binary format, like strings, styles, and the paths of images or layouts files, which are a part of this content. However, the data can only be processed in an XML format.

**Table 2:** Common android malware families.

Common android malware families					
Accu Track Ackposts	Counterclank Crusewind	FakeTaoBao FakeTimer	Kidlogger KMIN	Placms Plankton	SpyOO Ssucl
Acnetdoor	Dogowar	FakeUpdate/Apkqug	Ksapp	Podec	Steek/Fatakr
Adsms	Dougalek	Fakevertu	LeNa	PoisonCake	Tascudap
Airpush/StopSMS	DroidDeluxe	Find and Call/Fidall	Lien/	ProxyTrojan/NotCompatible/NioServ	TapSnake/ Droisnake
Anserver/Answerbot	DroidDream	Finspy	Locker/SLocker Ransomware	Qicsomos	TGloader/ Stiniter
Antares/	DroidJack/SandoRAT	Fjcon	Loicdos	Raden	TigerBot
Antammi Arspam AVpass BackFlash/Crosate	DroidDreamLight DroidKungfu Droidsheep	Flexispy Foncy Fokange/Fokonge	Loozfon Lovetrap/Luvrtrap Luckycat	Repane Roidsec/Sinpon RootSmart/ Bmaster	Tetus Titan Tonclank
Badaccents	DSEncrypt	Fonefee/Feejar	Maistealer	RuFraud	Tracer
Badnews	Extension/Monad	Gamex	Malap	Saiva	TypStu
BankBot Basebridge BeanBot	FaceNiff FakeAngry FakeApp.AL	Gazon Geinimi GGTracker	Mania MMarketPay MobiDash MobileSpy/Godwon	Samsapo Scavir Scipiex SaveMe/SocialPath	UpdtBot UpdtKiller Uracto
Beita	FakeAV	GingerBreak	MobileTx	Sndapps/Snadapps	USBcleaver
Binv	FakeDaum/Vmwol	GingerMaster/GingerBreaker	Mobinauten	SMSsniffer	Uten
BgServ	FakeBank	Godwon	Moghava	SpamBot	Uxipp
Biige	FakeDefender	GoldenEagle/GlodEagl	Nandrobox Netisend Nickispy Obad Oldboot/MouaBad OpFake	SeaWeth Selfmite Skullkey Smack SMSpacem SMSilence/SMSCatcher	Vdloader
Bosster Boxer Cajino Carberp Cawitt Code4hk/xRAT	FakeDoc FakeFlash FakeInst FakeJobOffer FakeMarket FakeMart	GoneIn60seconds GPspy HeHe Hidelcon HippoSMS HongTouTou/Adrd	PDAspy Penetho Photsy/Phopsy Pincer	SMSCatcher SMSreg Spitmo SMSspy SPPush	Walkinwat/Pirater Waps/Simhosy Wroba/HijackRAT YZHC Zeahache Zitmo/Citmo
Chulli Cellspy Coogos CopyCat Cosha	FakeNefix FakeNotify FakePlay FakePlayer FakeRegSMS	Iconosys Imlog Jifake JollyServ Jsmshider/Xsider	Pjapps	SpyBubble	ZergRush ZertSecurity Zsone

**Table 3:** Compare between static and dynamic analyses.

	Static	Dynamic
How it works	The suspected code is analyzed without the application being run during static analysis. This method involves disassembly of source code and analyzing it to check the presence of malware without executing the source code and depend only on malware abstraction characteristics and application byte code. Mostly, reengineering is applied [41–43].	The suspected code is analyzed during the runtime execution. It focuses on the characteristics and traces of suspicious use during implementation [24–26, 44–46]and also focuses on system calls and application programs. It is a cybernetic environment used for the execution of code.

Advantage	Harmful applications are not needed to be installed on the device.	It can detect dependencies that are impossible to detect in the static method.
	Do not execute or run the malware code.	Collects temporal instructions.
	Applications are in format APK or archive in a zip package [41–43].	Deals with real data, whereas. in the static analysis, you cannot know input files to be passed for analysis.
		It can overcome string detection issues, such as malware fitting and pleomorphism [41–43].

Disadvantage	This technique does not take into consideration the analysis of unknown malware.	Can have a negative performance impact on the application.
	The source codes used are not directly available, and it must be disassembled to extract the features [16–21].	Requires better mobile security at critical monitoring stages.
	Harmful applications cannot appear until the code has been run.	It can give incorrect results for similar behavior of the malicious applications with staring applications.
	Suffers from code obfuscation [9, 17, 22, 23].	It is a complex and time-consuming technique that requires high resource usage and storage capacity [22, 47].

**Table 4:** Various malware datasets' publication counts.

Dataset	Number of publications
Drebin	20
Repository	8
Collection	6
MalGenome	17

**Table 5:** Fixed image width according to the file size.

File size	Width
<50 kB	64
50 kB–100 kB	128
100 kB–200 kB	256
200 kB–500 kB	512
500 kB–1000 kB	1024

**Table 6:** Various combinations and its associated instances used in the study.

Combination	CR	AM	RS	CL	CR + AM	CR + RS	CR + CL	AM + RS	AM + CL	RS + CL	CR + AM + RS	CR + AM + CL	CR + RS + CL	AM + RS + CL	CR + AM + RS + CL
No. of instances	1826	4659	4659	4660	4659	4659	4660	4659	4660	4660	4659	4660	4660	4660	4660

**Table 7:** Generic and augmented CNN accuracies on 15 different grayscale malware image combinations.

	Image combination	CNN (%)	CNN-SVM (%)	CNN-KNN (%)	CNN-RF (%)	VGG16 (%)	GoogLeNet (%)	ResNeXt (%)	Modified ResNeXt (%)
1	CR	83.58	82.92	77.11	83.42	78.27	88.86	92.96	98.25
2	AM	89.79	90.18	83.94	84.85	85.76	90.76	92.51	95.50
3	RS	86.86	88.56	86.02	84.53	82.12	89.37	95.21	96.50
4	CL	89.46	90.57	89.40	87.58	87.23	91.16	94.74	95.63
5	CR + AM	91.48	92.59	86.93	87.52	90.57	89.81	92.74	96.88
6	CR + RS	87.12	89.47	86.80	85.89	88.91	89.16	94.08	97.38
7	CR + CL	89.33	90.25	89.01	88.43	89.34	90.01	93.85	96.94
8	AM + RS	88.29	89.47	87.78	84.98	86.78	90.07	93.86	96
9	AM + CL	89.33	90.83	89.79	88.69	84.43	90.07	92.06	95.57
10	RS + CL	88.49	90.96	89.34	87.58	84.37	85.77	94.98	96.07
11	CR + AM + RS	89.46	90.77	88.75	85.50	87.67	89.66	93.56	96.75
12	CR + AM + CL	89.33	90.51	88.49	88.82	86.81	90.26	93.40	96.46
13	CR + RS + CL	89.53	90.90	89.66	88.17	84.56	89.80	94.30	96.49
14	AM + RS + CL	88.55	90.70	89.86	87.97	89.29	90.43	94.15	95.88
15	CR + AM + RS + CL	89.33	90.70	89.60	87.84	84.32	90.04	93.86	96.47

**Table 8:** A comparison of execution time and images processed per second by the proposed model.

S/no.	Combination	Execution time (s)	Images processed/second
1	CR	231.2	6.57
2	AM	663.8	5.1
3	RS	787.4	4.25
4	CL	1102.1	4.21
5	CR + AM	790.2	4.23
6	CR + RS	1004.4	4.64
7	CR + CL	1109.7	4.2
8	AM + RS	850.5	4.34
9	AM + CL	1120.4	4.12
10	RS + CL	1093.3	4.26
11	CR + AM + RS	624.7	5.04
12	CR + AM + CL	1139.4	4.04
13	CR + RS + CL	1235.5	3.78
14	AM + RS + CL	1203.9	3.83
15	CR + AM + RS + CL	1513.7	3.08

**Table 9:** Confusion matrix for the top 20 malware families in the proposed model.

	FakeInstaller	DroidKungFu	Plankton	OpFake	GinMaster	BaseBridge	Iconosys	Kmin	FakeDoc	Geinimi	Adrd	DroidDream	ExploitLinuxLotoor	Mobile Tx	Glodream	FakeRun	SendPay	Gappusin	Imlog	SMSreg
FakeInstaller	904	0	0	17	0	0	1	0	0	1	0	0	0	0	0	0	0	0	0	2
DroidkungFu	0	579	3	2	13	10	0	0	0	0	34	0	6	0	3	0	0	17	0	0
Plankton	1	3	573	0	4	20	0	0	0	11	11	1	0	0	1	0	0	0	0	0
OpFake	0	0	0	560	51	0	0	0	0	0	0	0	0	0	2	0	0	0	0	0
GinMaster	0	1	2	3	315	0	0	0	0	1	12	0	0	0	4	0	0	1	0	0
BaseBridge	0	5	0	1	1	316	0	0	0	0	3	0	0	0	4	0	0	0	0	0
Iconosys	0	0	0	0	0	0	152	0	0	0	0	0	0	0	0	0	0	0	0	0
Kmin	0	0	0	0	0	0	0	135	0	0	12	0	0	0	0	0	0	0	0	0
FakeDoc	3	0	0	0	2	0	0	0	120	0	2	0	0	0	4	0	0	1	0	0
Geinimi	0	0	0	0	3	2	0	0	0	86	1	0	0	0	0	0	0	0	0	0
Adrd	0	1	0	0	1	1	0	0	0	0	88	0	0	0	0	0	0	0	0	0
DroidDream	0	1	0	0	0	0	0	0	0	0	1	78	0	0	0	0	0	1	0	0
ExploitLinuxLotoor	0	1	0	0	3	4	0	0	0	0	1	0	60	0	0	0	1	0	0	0
Mobile Tx	0	0	0	0	0	0	0	0	0	0	0	0	0	69	0	0	0	0	0	0
Glodream	0	2	0	1	1	1	1	0	0	0	2	0	0	0	60	0	0	0	0	0
FakeRun	0	0	21	1	0	0	0	0	1	0	3	0	1	0	4	27	0	3	0	0
SendPay	0	0	0	0	0	0	0	0	0	0	0	0	0	0	0	0	59	0	0	0
Gappusin	0	3	0	0	1	2	0	0	0	0	0	0	0	0	0	0	0	51	0	0
Imlog	0	0	0	0	0	0	0	0	0	0	0	0	0	0	0	0	0	2	41	0
SMSreg	0	0	1	0	0	0	0	0	0	1	0	0	0	0	0	0	0	0	0	39

**Table 10:** F1-score comparisons between the modified ResNeXt and the original ResNeXt in the Drebin dataset.

Family	ResNeXt	Modified ResNeXt
Adrd	0.67433	0.908108
BaseBridge	0.921283	0.961832
DroidDream	0.962963	0.981132
DroidKungFu	0.916865	0.935737
ExploitLinuxLotoor	0.875912	0.827068
FakeDoc	0.948617	0.988593
FakeInstaller	0.613636	0.99675
FakeRun	0.761194	0.97561
Gappusin	0.858311	0.866667
Geinimi	0.794702	0.891192
GinMaster	0.993464	0.939691
Glodream	0.97619	0.78481
Iconosys	0.957447	0.996721
Imlog	1	0.988506
Kmin	0.934891	1
Mobile Tx	0.93551	1
OpFake	0.991597	0.995938
Plankton	0.95122	0.994378
SMSreg	0.986361	0.886076
SendPay	0.895833	0.944

**Table 11:** Stability classification performance of the proposed model for the Drebin and AMD datasets.

Dataset	Precision	Recall	Accuracy
Drebin + Drebin	97.1	97.3	98.2
Drebin + S-AMD	66.2	67.3	66.2
Drebin + T-AMD	75.2	77.8	77.4
S-AMD + Drebin	87.1	87.2	89.1
S-AMD + S-ADM	83.3	88.1	83.5
T-AMD + Drebin	86.3	87.6	87
T-AMD + T-ADM	93	92.5	91.3

## Data Availability

The datasets used to support the findings of this study are included within the article.
